The article "Effects of Camrelizumab Combined with First-Line Chemotherapy on Serum SCC, VEGF Levels, and Adverse Reactions in Patients with Advanced Squamous Cell Carcinoma of the Lung" was retracted in 2023. Reasons: signs of a paper mill; suspected computer-generated content; unreliable results or conclusions; lack of ethics approval or compliance.

# Effects of Camrelizumab Combined with First-Line Chemotherapy on Serum SCC, VEGF Levels, and Adverse Reactions in Patients with Advanced Squamous Cell Carcinoma of the Lung

**DOI:** 10.1155/2022/3137370

**Published:** 2022-11-18

**Authors:** Zizong Wang, Yunpeng Xuan, Yanmei Shao, Qiang Zou, Hong Cui, Xiangfeng Jin

**Affiliations:** ^1^Department of Thoracic Surgery, The Affiliated Hospital of Qingdao University, Qingdao 266003, China; ^2^Department of Respiratory and Critical Care Medicine, The Affiliated Hospital of Qingdao University, Qingdao 266000, China; ^3^Department of Blood Transfusio, The Affiliated Qingdao Hiser Hospital of Qingdao University (Qingdao Hospital of Traditional Chinese Medicine), Qingdao 266000, China; ^4^Operation Room, The Affiliated Hospital of Qingdao University, Qingdao 266003, China

## Abstract

**Objective:**

To study the effects of camrelizumab accompanied by first-line chemotherapy on serum SCC, VEGF levels, and adverse reactions in people undergoing advanced lung squamous cell carcinoma.

**Methods:**

Data sources of the study subjects were 60 people suffering from advanced squamous cell carcinoma of the lung hospitalized from January 2018 to October 2019. They were assigned to two groups, including the control group and the observation group in a random manner, and each consisted of 30 patients. Those in the observation group received camrelizumab (SHR-1210), and gemcitabine plus cisplatin (GP) chemotherapy were treated in the control group. Finally, according to the results, we compare the data of patients in both groups so as to find out the similarities and differences.

**Results:**

Among them, the effective efficiency of clinical treatment in the control group reached 36.67%, and that in the observation group reached 56.67%. Intuitively, it can be concluded that the control group showed lower results than the observed group. The observed group turned out to have higher periodic survival and progression free survival (PFS) of patients than the other group. During and after the cycle treatment, the data of SCC and VEGF were reduced to some extent, but the control group appeared to have a more evident reduction rate than the other group.

**Conclusion:**

SHR-1210 combined with chemotherapy has a considerable effect in practical application and has excellent clinical performance.

## 1. Introduction

Lung squamous cell carcinoma is a unique pathological type, which can cause obstructive pneumonia and bronchial stenosis, seriously threatening human health and reducing life progress and quality index [1]. Squamous lung cancer is mostly found in the elderly male population, and its specific pathogenesis is not completely clear. But it is closely related to smoking history, genetics, atmospheric pollution, and ionizing radiation [2]. In the early stage of the disease, it was found that after certain treatment, the patient's physical quality and future life will be greatly improved. The early and middle stages of lung squamous carcinoma are mainly treated by surgery with a good prognosis. But advanced patients are treated mainly with chemotherapy. The growth of lung squamous cells is relatively slow, and there is no obvious response and hormone level change in the early stage. Patients generally enter the advanced stage when they are found [3, 4]. So how to effectively treat late stage lung squamous carcinoma has become one of the important problems faced today.

The article "Effects of Camrelizumab Combined with First-Line Chemotherapy on Serum SCC, VEGF Levels, and Adverse Reactions in Patients with Advanced Squamous Cell Carcinoma of the Lung" was retracted in 2023. Reasons: signs of a paper mill; suspected computer-generated content; unreliable results or conclusions; lack of ethics approval or compliance.

## 2. Literature Review

At present, gemcitabine and cisplatin (GP) are the first-line chemotherapy for squamous lung cancer, which can significantly enhance clinical efficacy and prolongs survival. But it does not achieve clinically satisfactory results [5]. Camrelizumab (SHR-1210) as an inhibitor, it can block the ligand pathway of PD-1 by binding PD-1, thus stimulating the recovery of antitumor immunity in the body and finally establishing the basic framework of immunotherapy [6, 7]. In the existing studies, SHR-1210 combined with chemotherapy can greatly change the living status of patients [8], but there are few combined therapies for lung squamous cell carcinoma, which has a certain research value. At present, no study has explored the effect of SHR-1210 combined with chemotherapy on the treatment effect of advanced lung squamous cell carcinoma from SCC and VEGF levels.

Therefore, this study intends to analyze the effects of SHR-1210 combined with chemotherapy on SCC and VEGF levels, cyclic survival rate, progression free survival (PFS), and adverse reaction rate in advanced lung squamous cell carcinoma at the clinical level, so as to provide a better data model for the clinical treatment of advanced lung squamous cell carcinoma.

## 3. Materials and Methods

### 3.1. Materials

The data sources for this study were 60 people suffering from advanced squamous cell carcinoma of the lung hospitalized from January 2018 to October 2019. Patients were assigned to two groups in a random manner, including the control group and the observation group, and each consisted of 30 subjects. Control group: GP chemotherapy regimen, observation group: GP + SHR-1210 chemotherapy regimen. The hospital committee has given approval to the study and the registration number is 110370000030426.

Some data of patients were not statistically significant and were only used as a reference for duplicate data.  Table 1 shows that there was no significant difference between the control group and the observation group in terms of gender (*P* = 0.887), age (*P* = 0.708), smoking (*P* = 0.492), and clinical stage (*P* = 0.501), indicating that later studies excluded the influence of confounding factors.

The article "Effects of Camrelizumab Combined with First-Line Chemotherapy on Serum SCC, VEGF Levels, and Adverse Reactions in Patients with Advanced Squamous Cell Carcinoma of the Lung" was retracted in 2023. Reasons: signs of a paper mill; suspected computer-generated content; unreliable results or conclusions; lack of ethics approval or compliance.

### 3.2. Criteria of Inclusion and Exclusion

Inclusion criteria are as follows [9, 10]:

1. . All patients undergoing intermediate and advanced lung squamous cell carcinoma by relevant diagnostic techniques
2. Receiving treatment for the first time
3. Normal body function
4. The patient and his family agreed to the treatment

Exclusion criteria are as follows [9, 10]:

1. Patients with drug allergy and chemotherapy allergy in this study
2. Patients who have taken other inhibitors
3. Patients with other complicated cancers
4. Those who quit halfway
5. Pregnant or midway pregnant

### 3.3. Patient Treatment

The control group received a GP chemotherapy regimen: gemcitabine 1000 mg/m2 intravenously on the first and eighth days and cisplatin 70 mg/m^2^ intravenously every 3 days. The observation group was additionally given SHR-1210, 200 mg intravenously every 3 weeks. 3 weeks was a cycle, and both groups were treated for 4 consecutive cycles.

### 3.4. Indicators

#### 3.4.1. Efficacy Evaluation

Complete remission (CR) is defined as the absence of lesions in a minimum of one month according to the response evaluation criteria in solid tumors (RECISTs) [11]. Partial remission (PR) is defined as a reduction in lesion area by at least 50% for a minimum of one month. Stable disease (SD) is defined as a lesion area reduction of less than 50% or an increase of 25% or less in a minimum of one month. PD is defined as at least a 50% reduction in lesion area or a 25% or less increase in lesion area for at least one month. PR means at least a 50% reduction in lesion area for a minimum of one month. SD means less than 50% reduction or an increase of 25% or less in lesion area in a minimum of one month overall clinical efficacy is expressed as CR and PR.

#### 3.4.2. Survival Rate and PFS

We observed subjects for one year in order to figure out the 1-year survival rate in both groups and to record the PFS (starting at the randomization group and ending at the time of first cancer progression or death) in both groups.

#### 3.4.3. Serum SCC and VEGF Levels

3 mL of venous blood from the fasting elbow was drawn from two groups of subjects 1 day prior to and 2 days following 4 cycles of treatment. The blood specimens were placed in EP tubes and rested for 1 h at room temperature, then they were centrifuged at 3000 rpm for 10 min with a VM-1400-2 KB centrifuge to separate the serum and stored at −80°C for measurement. Serum SCC levels and VEGF levels were measured by enzyme-linked immunosorbent assay (ELISA), and the kits used were provided by Sophia Biotechnology Co.

The article "Effects of Camrelizumab Combined with First-Line Chemotherapy on Serum SCC, VEGF Levels, and Adverse Reactions in Patients with Advanced Squamous Cell Carcinoma of the Lung" was retracted in 2023. Reasons: signs of a paper mill; suspected computer-generated content; unreliable results or conclusions; lack of ethics approval or compliance.

#### 3.4.4. Adverse Reactions

The occurrence of adverse reactions is observed such as thrombocytopenia, leukopenia, gastrointestinal reactions, liver and kidney injury, and bone marrow suppression in both groups.

### 3.5. Statistics

We have used the statistical analysis software SPSS 23.0. In this study to analyze data. Count data were presented as cases (*n*) or percentages (percent). Data of measurement were presented as mean standard deviation (s), *t*-test; *P* < 0.05 indicates that it was of great importance in statistics. The statistical results were then visualized using GraphPad 8.0.

## 4. Results

### 4.1. Comparison of the Clinical Efficacy of Two Groups

By analyzing the CR, PR, SD, and PD values of the two groups, compared to the observation group, the control group showed a notably lower clinical efficacy (*P* < 0.05) as shown in Table 2.

### 4.2. Comparison of 1-Year Survival Rate and PFS of Two Groups

Table 3 shows that the observed group turned out to have a notably higher 1-year survival rate than the control group and also have a great loner PFS than the other group, which is of great importance in statistics (*P* < 0.05).

### 4.3. Comparison of Serum SCC and VEGF Levels before and after Treatment between the Two Groups

Before they were given treatment, no statistically striking difference was found in serum SCC and VEGF levels between these two groups (*P* > 0.05). But following treatment, both groups showed a notably lower serum SCC and VEGF levels, with the observed group significantly lower than the other group.  Table 4 and Figure 1 show that the difference was of great importance in statistics (*P* < 0.05).

### 4.4. Comparison of Bad Reactions of Two Groups

As shown in Table 5, the difference in the occurrence of bad reactions of the two groups was of no importance in statistics (*P* > 0.05).

## 5. Discussion

Squamous lung cancer, advanced squamous lung cancer in particular, has a very high incidence and mortality rate in clinical practice and should be given great clinical attention [12]. As a first-line chemotherapy regimen for squamous lung cancer, GP can improve the quality of patient survival to some extent. However, patients' benefit is limited [13]. Recently, immune checkpoint inhibitors (ICIs) have been extensively applied to treat oncological illnesses in clinical practices because of their well-tolerated and growth advantages, allowing for breakthroughs in clinical practice. They can effectively prolong the life of patients [14, 15]; SHR-1210 is one of the familiar ICIs [16]. However, few research studies have investigated serum SCC and VEGF levels in people who suffer from advanced squamous lung cancer and whether adverse effects can be influenced by their combination with chemotherapy in the first-line. The results of this study found that SHR-1210 combined with chemotherapy first-line treatment could effectively down-regulate levels of serum SCC and VEGF in people undergoing advanced squamous lung cancer without increasing adverse effects. The reasons are analyzed as follows.

The article "Effects of Camrelizumab Combined with First-Line Chemotherapy on Serum SCC, VEGF Levels, and Adverse Reactions in Patients with Advanced Squamous Cell Carcinoma of the Lung" was retracted in 2023. Reasons: signs of a paper mill; suspected computer-generated content; unreliable results or conclusions; lack of ethics approval or compliance.

Liu and colleagues [17] investigated the efficacy of SHR-1210 accompanied by sorafenib in people undergoing advanced hepatocellular carcinoma. The findings of the study revealed that the combination of SHR-1210 and sorafenib was more effective than sorafenib alone; Lan and colleagues [18] discovered that the objective response rate of people who suffered from advanced cervical cancer and received SHR-1210 combined with apatinib reached 55.6 percent, and the median PFS is 8.8 months. The observation group turned out to have 56.67% of overall clinical efficiency, 60.00% of 1-year survival rate, and (8.241.42) months of PFS in the study, all notably higher than the other group. The findings are essentially in agreement with Liu and Lan's study, which suggests that treatment of advanced squamous lung cancer with SHR-1210 combined with chemotherapy was significant. The reasons were that Gemcitabine in GP chemotherapy regimens is a pyrimidine broad-spectrum anticancer drug with a mechanism of action similar to that of cytarabine, which refers to the production of active substances under the action of thymidine kinases in the human body, such as gemcitabine triphosphate and gemcitabine diphosphate. These substances exert an inhibitory effect on ribonucleotide activity, which in turn reverses the normal negative feedback inhibition of thymidine kinase, causing a large accumulation of gemcitabine triphosphate, which breaks deoxyribonucleic acid (DNA) and promotes cancer cell death [19]. Cisplatin, a nonspecific cell cycle drug, exerts its antitumor effects mainly by damaging cancer cell DNA [20]. SHR-1210 is an immunoglobulin G4 (IgG4) monoclonal antibody. It can bind PD-1 to prevent PD-1/PD-L1 binding. In order to reactivate immune response, the immune escape pathway of tumor cells must be cut off. Therefore, the function of immune surveillance will gradually recover, and the function of T lymphocytes to recognize and kill tumor cells will also be improved. Thus, it can exert its antitumor effect [21]. The combination of the GP chemotherapy regimen with SHR-1210 acts synergistically, exerting antitumor effects from different mechanisms, respectively.

The article "Effects of Camrelizumab Combined with First-Line Chemotherapy on Serum SCC, VEGF Levels, and Adverse Reactions in Patients with Advanced Squamous Cell Carcinoma of the Lung" was retracted in 2023. Reasons: signs of a paper mill; suspected computer-generated content; unreliable results or conclusions; lack of ethics approval or compliance.

As a tissue-specific glycoprotein tumor marker for squamous carcinoma, the level of SCC increases along with the aggravation of squamous carcinoma, which has positive significance for clinical assessment of the efficacy, prognosis, and recurrence of squamous carcinoma patients [22]. VEGF is a provascular endothelial growth factor induced by hypoxia, which can increase vascular permeability by binding to vascular endothelial cell receptors, induce endothelial cell proliferation as well as promote stromal lysis and inflammatory exudation, and accelerate the proliferation of tumor cells, therefore, the proliferation and differentiation of tumor cells can be reduced by inhibiting the expression of VEGF, which facilitates clinical treatment [23]. Ma [24] found that inhibition of VEGF expression could inhibit NSCLC angiogenesis. In this study, after a period of treatment, the levels of serum SCC and VEGF decreased in both groups, and the observed group showed lower levels than those in the other group. Ma's comprehensive research results show that the combination of SHR-1210 and chemotherapy in the first-line treatment of advanced squamous cell carcinoma can reduce the levels of serum SCC and VEGF. The reason for this is that SHR-1210 prevents the binding of programmed death ligand-2 (PD-L2) and PD-L1 through specific target binding with PD-1, which in turn enhances the immune response by improving the body's immune function. SHR-1210 also reduces the proportion of oxygen-depleted cells in tumors, promotes increased oxygenation, and directly improves radiosensitivity, promotes apoptosis, reduces tumor neovascularization, and then effectively down-regulates serum SCC and VEGF levels in cancer patients [25].

Zhang [26] found that on the basis of radiotherapy, the toxicity of SHR-1210 in people undergoing locally advanced esophageal squamous cell carcinoma was controllable; in this study, in general agreement with Zhang's findings, no notable difference was found in the occurrence of various bad reactions between two groups, implying that there is no increased risk of adverse reactions with SHR-1210 combination chemotherapy in the first-line treatment of advanced squamous carcinoma. The reason for this is that SHR-1210 has the potential to cause some immune-related adverse reactions, causing the involvement of several systems such as the liver, endocrine, and skin; however, it has been shown in relevant studies that combining it with chemotherapy help effectively lower its occurrence [25].

The limitation of this research is the sample size selected is small, which may cause discrepancies between the data in the results and the actual values, so the sample size needs to be expanded. In addition, this study only initially explored the effect of camrelizumab combined with first-line chemotherapy on serum SCC, VEGF levels, and adverse reactions in patients with advanced lung squamous cell carcinoma, and further experiments will be conducted to explore its specific treatment mechanism in the later stage.

The article "Effects of Camrelizumab Combined with First-Line Chemotherapy on Serum SCC, VEGF Levels, and Adverse Reactions in Patients with Advanced Squamous Cell Carcinoma of the Lung" was retracted in 2023. Reasons: signs of a paper mill; suspected computer-generated content; unreliable results or conclusions; lack of ethics approval or compliance.

## 6. Conclusion

In conclusion, SHR-1210 and chemotherapy in the first line can effectively improve the clinical outcome of advanced squamous lung cancer, increase survival rate and prolong survival, and also reduce serum SCC and VEGF levels, at the same time, the risk of adverse reactions does not remain decreased. This is a very worthwhile reference in clinical medicine.

## Figures and Tables

**Figure 1:** Comparison of serum SCC and VEGF levels of two groups before and after they received treatment. Note: ^*∗*^*P* < 0.05 compared with pretreatment; ^#^*P* < 0.05 compared with the control group.

**Table 1:** Comparison of two groups of data.

Materials		Control group (*n* = 30)	Observation group (*n* = 30)	*t*/*χ*^2^	*P*
Gender	Male	25 (83.33)	24 (80.00)	0.023	0.887
	Female	5 (16.67)	6 (20.00)		

Average age		56.02 ± 7.07	55.50 ± 7.14	0.372	0.708

Smoking history	Yes	27 (90.00)	26 (86.67)	0.473	0.492
	No	3 (10.00)	4 (13.33)		

Clinical stages [*n* (%)]	?	6 (20.00)	8 (26.67)	0.454	0.501
	IV	24 (80.00)	22 (73.33)		

**Table 2:** Comparison of clinical efficacy of two groups [*n* (%)].

Clinical efficacy	Control group (*n* = 30)	Observation group (*n* = 30)	*χ* ^2^	*P*
CR	0 (0.00)	0 (0.00)	—	—
PR	11 (36.67)	17 (56.67)	—	—
SD	8 (26.67)	8 (26.67)	—	—
PD	11 (36.67)	5 (16.67)	—	—
Total clinical effectiveness	11 (36.67)	17 (56.67)	5.689	0.027

**Table 3:** Comparison of 1-year survival rate and PFS of two groups.

Project	Control group (*n* = 30)	Observation group (*n* = 30)	*t*/*χ*^2^	*P*
Survival rate [*n* (%)]	9 (30.00)	18 (60.00)	6.214	0.018
PFS (month)	6.33 ± 1.21	8.24 ± 1.42	7.062	0.009

**Table 4:** Comparison of serum SCC and VEGF levels between the two groups before and after they received treatment ($\bar{x}$ ±*s*).

Indicators		Control group (*n* = 30)	Observed group (*n* = 30)
SCC (ng/L)	Before treatment	40.13 ± 5.06	40.01 ± 5.02
	After treatment	28.71 ± 3.07^*∗*^	21.40 ± 2.74^*∗*^^#^

VEGF (pg/mL)	Before treatment	608.23 ± 68.21	609.34 ± 69.66
	After treatment	471.58 ± 42.31^*∗*^	334.59 ± 38.72^*∗*^^#^

*Note.* ^*∗*^ *P* < 0.05 compared with that before treatment; ^#^*P* < 0.05 compared with the control group.

**Table 5:** Comparison of adverse reactions between the two groups [*n* (%)].

Adverse reactions	Control group (*n* = 30)	Observation group (*n* = 30)	*χ* ^2^	*P*
Thrombocytopenia	6 (20.00)	7 (23.33)	0.072	0.790
Leukopenia	6 (20.00)	5 (16.67)	0.206	0.651
Gastrointestinal reactions	10 (33.33)	8 (26.67)	0.398	0.528
Injuries of liver and kidney	7 (23.33)	7 (23.33)	0.000	1.000
Bone marrow suppression	5 (16.67)	4 (13.33)	0.165	0.685

The article "Effects of Camrelizumab Combined with First-Line Chemotherapy on Serum SCC, VEGF Levels, and Adverse Reactions in Patients with Advanced Squamous Cell Carcinoma of the Lung" was retracted in 2023. Reasons: signs of a paper mill; suspected computer-generated content; unreliable results or conclusions; lack of ethics approval or compliance.

## Data Availability

The data used to support the findings of this study are available from the corresponding author upon request.
